# Radiation mitigating properties of the lignan component in flaxseed

**DOI:** 10.1186/1471-2407-13-179

**Published:** 2013-04-04

**Authors:** Ralph Pietrofesa, Jason Turowski, Sonia Tyagi, Floyd Dukes, Evguenia Arguiri, Theresa M Busch, Shannon M Gallagher-Colombo, Charalambos C Solomides, Keith A Cengel, Melpo Christofidou-Solomidou

**Affiliations:** 1 Department of Medicine, Pulmonary, Allergy and Critical Care Division, University of Pennsylvania, 3615 Civic Center Boulevard, Abramson Research Building, Suite 1016C, Philadelphia, PA, 19104, USA; 2 Radiation Oncology, University of Pennsylvania Medical Center, Philadelphia, PA, 19104, USA; 3 Department of Pathology, Jefferson University Hospital, Philadelphia, PA, 19104, USA

**Keywords:** Flaxseed lignan complex, Radiation pneumonopathy, Radiation dispersion device, Mitigation, Lung fibrosis, Antioxidant, Nitrotyrosine, TBARS, TGF-beta 1, SDG, SARRP, ROS

## Abstract

**Background:**

Wholegrain flaxseed (FS), and its lignan component (FLC) consisting mainly of secoisolariciresinol diglucoside (SDG), have potent lung radioprotective properties while not abrogating the efficacy of radiotherapy. However, while the whole grain was recently shown to also have potent mitigating properties in a thoracic radiation pneumonopathy model, the bioactive component in the grain responsible for the mitigation of lung damage was never identified. Lungs may be exposed to radiation therapeutically for thoracic malignancies or incidentally following detonation of a radiological dispersion device. This could potentially lead to pulmonary inflammation, oxidative tissue injury, and fibrosis. This study aimed to evaluate the radiation mitigating effects of FLC in a mouse model of radiation pneumonopathy.

**Methods:**

We evaluated FLC-supplemented diets containing SDG lignan levels comparable to those in 10% and 20% whole grain diets. 10% or 20% FLC diets as compared to an isocaloric control diet (0% FLC) were given to mice (C57/BL6) (n=15-30 mice/group) at 24, 48, or 72-hours after single-dose (13.5 Gy) thoracic x-ray treatment (XRT). Mice were evaluated 4 months post-XRT for blood oxygenation, lung inflammation, fibrosis, cytokine and oxidative damage levels, and survival.

**Results:**

FLC significantly mitigated radiation-related animal death. Specifically, mice fed 0% FLC demonstrated 36.7% survival 4 months post-XRT compared to 60–73.3% survival in mice fed 10%-20% FLC initiated 24–72 hours post-XRT. FLC also mitigated radiation-induced lung fibrosis whereby 10% FLC initiated 24-hours post-XRT significantly decreased fibrosis as compared to mice fed control diet while the corresponding TGF-beta1 levels detected immunohistochemically were also decreased. Additionally, 10-20% FLC initiated at any time point post radiation exposure, mitigated radiation-induced lung injury evidenced by decreased bronchoalveolar lavage (BAL) protein and inflammatory cytokine/chemokine release at 16 weeks post-XRT. Importantly, neutrophilic and overall inflammatory cell infiltrate in airways and levels of nitrotyrosine and malondialdehyde (protein and lipid oxidation, respectively) were also mitigated by the lignan diet.

**Conclusions:**

Dietary FLC given early post-XRT mitigated radiation effects by decreasing inflammation, lung injury and eventual fibrosis while improving survival. FLC may be a useful agent, mitigating adverse effects of radiation in individuals exposed to incidental radiation, inhaled radioisotopes or even after the initiation of radiation therapy to treat malignancy.

## Background

Ionizing radiation can cause deleterious effects in living organisms. Technological advancement has increased human exposure to ionizing radiation through diagnostic and therapeutic radiographic procedures, as well as through daily workplace activities [1]. Humans are also exposed to ionizing radiation above background levels during air and space travel, from nuclear accidents, and through the use of electronic devices. Additionally, global developments over the past decade have established terrorism as a novel and highly concerning means by which large numbers of people could be exposed to potentially lethal amounts of radiation [2].

There are at least two potential ways that a terroristic attack could expose a population to radiation injury. If terrorists gained possession of a nuclear warhead, detonation could release large amounts of radiation (in a single “blast”) that could induce radiation sickness, bone marrow damage, and potential lung injury. More likely, the weapon of radiological terrorism would be a “dirty bomb,” or a radiological dispersion device (RDD). Conventional explosives would spread radioactive materials in the form of powder or pellets [2-4] that could spread far away from the immediate explosion and pose a significant health risk if inhaled. Whole-body irradiation induces acute radiation syndrome (ARS) with symptoms caused by damage to the hematopoietic, gastrointestinal and central nervous systems [5]. The lung becomes the target organ for radiation injury from an RDD.

Radiation pneumonopathy is defined as a significant clinical toxicity from thoracic radiation [6,7]. Patients receiving large doses of radiation to the lung demonstrate two adverse clinical scenarios [8]. An acute type of toxic radiation response can occur within weeks after irradiation followed by a second type of radiation-induced lung injury which can begin within several months after exposure; This is characterized as the “late fibrotic” phase, in which the number of inflammatory cells (particularly neutrophils) decrease and a marked thickening of alveolar walls due to collagen deposition can be noted histopathologically [9,10]. Radiation pneumonopathy has been modeled in animals [9]; C57/BL6 mice are especially susceptible to this fibrotic reaction [11-13].

Several agents, ranging from cytokines to receptor blockers, have been tested for their efficacy in ameliorating radiation effects [12,14-16]. Most agents, even those proven to be effective as radioprotectors (administered prior to a radiation exposure) unfortunately are not yet available for human use. These agents were intended as treatments for radiation injuries resulting from the therapeutic use of radiation — a very different scenario compared to radiation injuries resulting from nuclear accidents or radiological terrorism. In most accidental or terrorism scenarios 1) treatment would not be initiated until after the irradiation, thus eliminating agents that work only when given before irradiation; 2) radiation would be received in a short time frame and agents effective in multi-week radiation treatments might be less effective for a single large dose of radiation; and 3) a mitigator would need to be administered to a large population of healthy individuals exposed to an undetermined dose of radiation. Therefore, it has become highly desirable to find an agent that is non-toxic, cost-effective, and safe for multiple administrations with beneficial effects spanning a long radiation exposure and post-radiation exposure recovery phase.

Significant systemic toxicity associated with chemical radioprotectors [17,18] has shifted the focus to plants, herbs, as well as antioxidant agents to evaluate their radioprotective potential [19]. Our group has identified flaxseed (FS) and its bioactive lignan component (FLC) as potent protectors against radiation-induced lung injury when given prior to radiation exposure [20-22]. Specifically, dietary FS decreased radiation-induced oxidative lung tissue damage, decreased lung inflammation and prevented lung fibrosis. Our previous work demonstrated that FS given after thoracic radiation mitigated radiation effects by decreasing cytokine release, inflammation, and pulmonary fibrosis while improving mouse survival [22]. We also recently showed that FS has also potent radiation mitigating properties [22]. Our study of the whole grain, however, did not allow for the identification of the bioactive ingredient of FS that mediated radioprotective- and radiation-mitigating properties. We further designed studies that provided the first evidence that FLC, the lignan component in FS enriched in the phenolic, secoisolariciresinol diglucoside (SDG) surpassed whole grain FS in terms of antioxidant, anti-inflammatory and anti-fibrotic properties [20] and was indeed responsible for the radioprotective properties of the whole grain. However, the radiation mitigating effects of FLC (and the lignan SDG more specifically) were never investigated. The current study was performed to ascertain whether FLC, in addition to its radioprotective properties, could also be an effective mitigator of radiation toxicity when administered at different time points soon after radiation exposure to the lung. Evidence provided in this study provides novel, strong support that the bioactive ingredient in whole grain FS responsible for its radiation mitigating properties is the lignan component and more specifically SDG. Focusing on SDG as a radiation mitigator will allow detailed mechanistic studies in the future and further development into a drug with clinical usefulness thus showing how from a natural product and a common botanical, a chemical agent can be identified with enormous clinical implications.

## Methods

### Animals

Our studies used female C57/BL6 mice, a strain well characterized in the field of pulmonary radioprotection [23-25]. Mice were obtained from Charles River (Wilmington, MA) and irradiated at 6–8 weeks of age under animal protocols approved by the Institutional Animal Care and Use Committee (IACUC) of the University of Pennsylvania. Animals were housed in conventional cages under standardized conditions with controlled temperature and humidity and a 12:12-hour day-night light cycle. Animals had free access to water and formulated study diets. For this study we used n=15-30 mice for each irradiated (XRT, 13.5Gy) group (0% FLC, 10% FLC, and 20% FLC).

### Diet composition and dietary treatments

Three diets were used for this study, all based on a semi-purified AIN-93G diet which was modified to contain the test ingredient as previously described [20]. Importantly, control (no test ingredient added) and experimental diets were isocaloric, isonitrogenous, and contained equal amounts of dietary lipid and carbohydrate. Diets contained flaxseed lignan complex (FLC) at three different concentrations (0%, 10%, and 20%). These concentrations reflect amounts of the main FS lignan SDG comparable to those found in 0%, 10%, and 20% whole grain FS diets. The FLC, enriched in the lignan SDG (35% SDG content) was kindly provided by Archer Daniels Midland Inc., (ADM, IL). Mice were maintained on control (0% FLC) diet given ad libitum for three days prior to XRT. 10% or 20% FLC diets were then started at 24, 48, and 72 hours post-XRT and continued for the duration of the study (Scheme, Figure 1). Control-fed mice remained on 0% FLC diet throughout the course of the study.

**Figure 1:** **Experimental plan of animal feeding protocol and radiation exposure.** Mice were pre-fed 0% FLC for 72 hours prior to single fraction thoracic X-ray radiation therapy (13.5 Gy). Following XRT exposure, mouse cohorts (n=15) were fed 10% FLC or 20% FLC diets initiated 24, 48, or 72 hours post-XRT. Control-fed mouse cohorts remained on 0% FLC diet throughout the course of the study. Mice were sacrificed at 16 weeks post-XRT.

### Analytical evaluation of FS lignan metabolite levels in murine plasma samples

Circulating plasma levels (Figure 2) of the flaxseed lignans enterodiol (ED) and enterolactone (EL) at time of sacrifice (16 weeks post-XRT) were determined by liquid chromatography tandem mass spectrometry (LC/MS/MS) as described earlier [13,21,26] using commercially available standards in 95% purity (Chromadex, Inc., Santa Ana, CA).

**Figure 2:** **Detection of flaxseed lignan metabolites enterodiol (ED) and enterolactone (EL) in plasma of mice fed FLC diets.** Circulating mammalian lignans, **Panel A**: enterodiol (ED) and **Panel B**: enterolactone (EL) levels in plasma of mice were determined using GC/MS/MS. Mouse cohorts were initiated on the control 0% FLC diet 3 days prior to XRT exposure. At 24 hours post-XRT 10% FLC and 20% FLC diets were initiated. Control-fed mouse cohorts remained on 0% FLC diet throughout the course of the study. Mouse cohorts were sacrificed at 16 weeks post-XRT and plasma was collected. Data is represented as mean ± SEM (n=5 mice / group). No statistical significance was found between XRT and no XRT.

### Radiation procedure

The Small Animal Radiation Research Platform (SARRP), (Xstrahl, Camberley, United Kingdom) was used to irradiate animals using a custom-made beam collimator. This system uses a Varian model NDI-225-22 kV x-ray tube mounted on a gantry that rotates between 0 and 120 degrees. The custom collimator creates a 12.5 cm circular field with well-defined borders and with animals arranged in a circular, “head in” arrangement (Figure 3) using a single central shield which provides uniform irradiation to the thoracic portion of multiple mice simultaneously. This set-up consists of a single, anterior 225kV, 15mA x-ray beam with a 0.15mm Cu at an SSD of 35cm that is designed to accurately reproduce the internal radiation dose distribution in mice that were used in previous studies [21,22,27]. The dosimetry and shielding of this system has been tested extensively [28]. The dose of radiation is a single fraction delivered via single AP (anterior-posterior) approach. The dose used is 13.5 Gy (roughly corresponding to LD50) as described in our previous work [12,21,27]. For quality assurance, thermoluminescent dosimeters are placed over selected mice, to verify correct dose administration.

**Figure 3:** **Irradiation of mouse thorax using the SARRP. Panel A**: Whole thorax irradiation jig and beam arrangement. **Panel B**: Radial arrangement of mice on platform. **Panel C**: Lead shielding of head area and upper extremities. **Panel D**: Lateral radiograph of mouse on the SARRP platform using thoracic irradiation jig. Mice were irradiated using the SARRP, to deliver single fraction 13.5 Gy X-ray irradiation to the thorax. Shielding was provided for the head only as the highly collimated field edge already limits dose to the abdomen/pelvis. The red shaded area represents the radiation field.

### Evaluation of cardiopulmonary function parameters

Prior to sacrifice, at 16 weeks post-XRT, pulse oximetry was performed, as previously described [20], on conscious mice (n=5/group) using a MouseOx non-invasive vital signs monitor (STARR Life Sciences Corp., Oakmont, PA). A mouse collar sensor was used to obtain measurements for arterial oxygen saturation (S_p_O_2_), pulse distension, respiratory rate, and heart rate. To minimize stress and maintain body temperature, mice were placed on a heating pad. Three minutes of continual readings were taken from each mouse and sorted in a spreadsheet using a macro that removed readings that reported any error codes. Subsequently, readings with no recorded error codes were averaged for each mouse and values reported as mean ± SEM for the total recording.

### Bronchoalveolar lavage fluid analysis

Mice were euthanized using an overdose of ketamine (100 mg/ ml) and xylazine (20 mg/ml) at 16 weeks post irradiation. Bronchoalveolar lavage (BAL) was then performed as described previously [12,21,27,29]. Briefly, BAL fluid was obtained using a 20-gauge angiocatheter (BD Pharmingen, San Diego, CA), with the intra-tracheal instillation of 1 ml phosphate-buffered saline (PBS) containing an anti-protease cocktail (Sigma) and 5 mM EDTA given in 0.5 ml increments [13,21,27]. An aliquot was immediately separated to measure total leukocyte cell counts (cells/ml BAL fluid) using a Coulter Cell and Particle Counter (Beckman Coulter, Miami, FL). The remaining lavage fluid was centrifuged at 1,200 rpm for 10 min and the cell-free supernatant was frozen at -80°C for cytokine determination, protein analysis, and evaluation of oxidative stress. The amount of total protein in the BAL fluid was assayed using the BCA Protein Assay Kit (Pierce, Rockford, IL) as per manufacturer’s instructions. Absorbance was read at 560 nm (MRX Microplate Reader, Dynatech Laboratories, Chantilly, VA) and protein levels in mg/ml of BAL fluid were calculated.

### Method for Measuring TBARS in BAL

BAL cytokine concentrations were determined, as previously described [22], using Invitrogen's Mouse Cytokine 20-Plex Panel (LMC0006). This multiplex panel permits simultaneous quantification of multiple cytokines in solution by capturing them onto antibody coated spectrally distinct fluorescent microspheres and measuring fluorescence intensity using the BioPlex 200 (Bio-Rad Laboratories, Hercules, CA) system. The assay was performed according to the manufacturer's protocol. All the samples were run in duplicate. The detection limit of this kit is in pg/ml for all the included cytokines.

### Multiplexed cytokine analysis of BAL

BAL cytokine concentrations were determined, as previously described [29], using Invitrogen's Mouse Cytokine 20-Plex Panel (LMC0006). This multiplex panel permits simultaneous quantification of multiple cytokines in solution by capturing them onto antibody coated spectrally distinct fluorescent microspheres and measuring fluorescence intensity using the BioPlex 200 (Bio-Rad Laboratories, Hercules, CA) system. The assay was performed according to the manufacturer's protocol. All the samples were run in duplicate. The detection limit of this kit is in pg/ml for all the included cytokines.

### Tissue harvesting, evaluation of pathology and quantitative measurement of fibrosis

The fibrosis endpoint for radiation experiments was 16 weeks post-XRT, corresponding to late radiation-induced fibrosis as readily detectable in our model [12,21,27] using biochemical assays and histopathological evaluation. The study aimed to specifically address the mitigation properties of FLC administered post-XRT exposure and the long-term benefits 16 weeks after initial exposure. For histological studies, the lungs prior to removal from the animal were instilled with 0.75 ml of buffered formalin through a 20-gauge angiocatheter placed in the trachea, immersed in buffered formalin overnight and processed for conventional paraffin histology. Sections were stained with hematoxylin and eosin and examined by light microscopy. Collagen content of mouse lung was evaluated quantitatively by determining hydroxyproline content using acid hydrolysis [12] according to Woessner *et al.*[30]. The data is expressed as μg hydroxyproline/whole lung. Semi-quantitative evaluation of fibrosis was done histologically by determining a radiation Fibrotic Index (FI) as described previously [21].

### Immunohistochemistry

Paraffin embedded lungs were sectioned and processed for routine immunohistochemistry as described earlier [12]. The following antibodies were used: anti-nitrotyrosine (rabbit polyclonal, a kind gift from Dr Harry Ischiropoulos, University of Pennsylvania, PA) [31]; anti-TGF-beta1, clone 1D11, (Genzyme Corp.) [32].

### Quantitative morphometric analysis of TGF- beta staining

Quantitative morphometric analysis of TGF- beta staining in lung tissues was performed on 5 μm serial lung sections stained with an antibody to TGF- beta1 (clone 1D11). Image analysis was performed using the Aperio ScanScope SC (Aperio Technologies, USA), Aperio ImageScope. Scanned slides were analyzed using the positive pixel count algorithm (version 8.1), by selection of threshold values for Iwp- high (the intensity threshold (upper limit) of weak positive pixels), Iwp-low (the intensity threshold (lower limit) of weak positive pixels) and Ip-low (the intensity threshold (lower limit) of medium positive pixels) that distinguished TGF-beta positive from unstained tissue. Threshold values were fixed across analysis of all sections. Data were quantified as the percent positive tissue, i.e. the number of strongly positive pixels (i.e. TGF-beta positive) relative to total tissue area (in pixels). Three images from all lung lobes were evaluated from each animal (n=3 mice per experimental cohort).

### Statistical analysis

Results are expressed as mean ± SEM of two independent experiments. Statistical differences among groups were determined using one-way analysis of variance (ANOVA). When statistically significant differences were found (*p*<0.05) individual comparisons were made using the Bonferoni/Dunn test (Statview 4.0). The survivor function was calculated using the Kaplan-Meier estimation method. Subsequently, Kaplan-Meier survival curves were generated using Stata data analysis and statistical software (release 12, Stata Corp, College Station, TX). Overall log-rank test for equality of survivor functions among mouse cohorts was performed. Subsequent post-hoc analysis between individual treatments was also performed.

## Results

### Dietary FLC was well tolerated over prolonged ingestion achieving biologically relevant levels

Mice tolerated FLC supplementation very well throughout the duration of the study. Prolonged feeding (>16 weeks) did not result in any differences in mouse weights among non-irradiated control groups fed FLC diets (data not shown). As a measure of diet palatability, no differences in feed intake were also noted. 0% FLC was compared with 10% and 20% FLC diets to confirm the physiological fuel values of treatment diets.

Circulating levels of the FS lignan metabolites enterolactone (EL) and enterodiol (ED) were quantified from the plasma of mice fed 0% FLC, 10% FLC and 20% FLC diets at 16 weeks post-XRT exposure. As expected, EL and ED were notably higher in groups fed 10% and 20% FLC compared to mice fed control, 0% FLC diet (Figure 2). Furthermore, a separate comparison was done to detect the difference at 16 weeks post-XRT in plasma lignan levels in irradiated vs non-irradiated mice fed 10% and 20% FLC diets (diets were initiated 24 hours post-XRT). ED in the mice fed FLC-fed, irradiated mice reached biologically relevant levels comparable to non-irradiated control mice fed the same diets and sacrificed at the same time (Figure 2A). EL was noticeably higher in irradiated mice fed 10% and 20% FLC at 24 hours post-XRT then sacrificed at 16 weeks (Figure 2B). Importantly, as anticipated, ED and EL levels in 10% FLC cohort were comparable to those we reported in our previous studies from feeding 10% wholegrain flaxseed [22] while those in the 20% FLC cohort were significantly 2-5-fold higher.

### Dietary FLC improved survival after thoracic radiation

We evaluated the effect of FLC diet on mitigating XRT-induced mortality in mice (Figure 4, A-C). The treatment diets (10% and 20% FLC) were started at three different time points soon after radiation exposure. As expected, the group fed the control diet and irradiated with 13.5 Gy showed a progressive pattern of XRT-induced mortality, comparable to previously published reports [20,21]. However, all FLC-fed mice showed improved survival rates as shown in Figure 4. Specifically, irradiated mice fed a 0% FLC diet had a survival rate of 36.7% at 16-weeks as compared to 60–73.3% survival in irradiated mice fed 10%-20% FLC diets initiated 24–72 hours post-XRT. Kaplan-Meier survival estimates were calculated for all animals involved in the study. The survival benefit with FLC diets was statistically significant with *p* values ranging from 0.01-0.05 as shown in the individual comparisons (Figure 4). This established FLC as a potent mitigator of radiation-induced mortality, as effective as the whole grain, shown in previous studies.

**Figure 4:** **Effect of FLC diets on the survival of mice through 16 weeks post-XRT.** Kaplan-Meier curves for overall survival. Mice were pre-fed 0% FLC for 72 hours prior to single fraction thoracic X-ray radiation therapy (13.5 Gy). Following XRT exposure, mouse cohorts (n=15) were fed 10% FLC or 20% FLC diets initiated **Panel A**: 24, **Panel B**: 48 or **Panel C**: 72 hours post-XRT and survival was observed up to 16 weeks post-XRT. Control-fed mouse cohorts remained on 0% FLC diet throughout the course of the study. No mice were lost in the non-irradiated cohorts (100% survival-not shown). Log-rank *p*-values (shown in figure) were calculated by log-rank test between irradiated mouse cohorts. Overall survival at 16 weeks post-XRT is depicted in the bar graph.

### Dietary FLC prevented lung injury, inflammation and improved blood oxygenation levels in mice 16 weeks post-XRT

Blood oxygenation saturation levels 16 weeks post-radiation exposure were measured in all mouse cohorts to extrapolate the extent of pneumonopathy from radiation exposure. Pulse oximetry was measured via a non-invasive sensor collar clip attached to each mouse. Figure 5A reveals the dose response of arterial oxygen saturation (SaO_2_) based on percent FLC administered post-XRT. Specifically, SaO_2_ of non-irradiated mice fed 0% FLC, 10% FLC or 20% FLC diet were compared at 16 weeks post-XRT to irradiated mice fed the same diets introduced at 24, 48, or 72 hours post-XRT (Figure 5A). Mice fed 10% FLC at 24 hours post-XRT had significantly higher (SaO_2_) at 16 weeks post-XRT (*p*≤ 0.01) compared with irradiated mice fed 0% FLC. Irradiated mice fed control diet had consistently lower average oxygen saturations ranging from the mid-to-high 80% range compared to FLC fed mice who mostly maintained average saturations in the mid-to-high 90% range. Remarkably, irradiated mice fed 10% FLC at 24 hours post-XRT had the highest average oxygen saturations overall. FLC shares similar radiation mitigating properties with the whole grain, in terms of protection of lung mechanics post-radiation exposure [22].

**Figure 5:** **Evaluation of blood oxygenation levels and lung injury in mice 16 weeks post-XRT.** Mice were pre-fed 0% FLC for 72 hours prior to single fraction thoracic X-ray radiation therapy (13.5 Gy). Following XRT exposure, mouse cohorts (n=15) were fed 10% FLC or 20% FLC diets initiated 24, 48, or 72 hours post-XRT. Control-fed mouse cohorts remained on 0% FLC diet throughout the course of the study. Mice were sacrificed at 16 weeks post-XRT. **Panel A**: Pulse oximetry analysis was performed prior to sacrifice at 16 weeks post-XRT. Data is represented as mean ± SEM. *p< 0.01 for irradiated 0% FLC vs. irradiated 10% FLC (+24 Hours). **Panel B**: BAL protein levels were determined at 16 weeks post-XRT. Data is represented as mean ± SEM. *p< 0.01 for irradiated 0% FLC vs. irradiated 10% and 20% FLC.

Radiation induced lung injury was evaluated by quantifying bronchoalveolar lavage (BAL) protein levels in all cohorts at 16 weeks post a single dose of thoracic XRT (Figure 5B). As anticipated, non-irradiated mice fed 0%, 10%, and 20% FLC diets showed negligible levels of BAL proteins. Irradiated mice fed 0% FLC demonstrated >3mg/ml BAL protein comparable to the injury shown in our previous studies [22]. Conversely, irradiated mice fed 10% and 20% FLC 24 post-XRT showed significantly lower (*p*<0.01) BAL protein levels, and thus, lung injury levels. Similarly, irradiated mice fed 10% FLC 48-hours post-XRT and irradiated mice fed 20% FLC 72-hours post-XRT had significantly lower levels of BAL protein compared to irradiated 0% FLC fed mice.

### Dietary FLC mitigated lung oxidative and nitrosative tissue damage induced by a single fraction of thoracic radiation

Increased nitrotyrosine production is associated with radiation-induced lung injury in rodent models [33]. We therefore evaluated lung sections for the presence of nitrotyrosine using immunohistochemisrty. As anticipated, nitrotyrosine staining of histological lung sections revealed intense positivity in sections from irradiated mice fed control diet. Staining was identified in the alveolar wall as well as in alveolar macrophages (Figure 6A, b). Importantly, positivity was low, almost undetectable in sections from irradiated lungs, from FLC-fed mice (Figure 6A, d,f).

**Figure 6:** **Oxidative and nitrosative stress in lung tissues 16 weeks post radiation exposure.** Mice on control diet (0% FLC) were exposed to a single fraction thoracic X-ray radiation therapy (13.5 Gy). Following XRT exposure, mice were switched to 10% FLC or 20% FLC diets that were initiated 24 hours post radiation exposure while control-fed mouse cohorts remained on 0% FLC diet throughout the course of the study. Lungs were harvested at 16 weeks post-XRT, and BAL performed followed by paraffin embedding and immunostaining for nitrotyrosine; brown staining (**Panel A**). Representative lung sections are shown In **Panels a-b:** representing 0% FLC, **Panels c-d:** representing 10% FLC and **Panels e-f:** representing 20% FLC. Sections were counterstained with methyl green. (Magnification 400X). Levels of thiobarbituric acid reactive substances (TBARS) in BAL samples were determined at 16 weeks post-XRT (**Panel B**). Data is represented as mean ± SEM. # *p*< 0.05 for 0% FLC vs. irradiated 0% FLC; *p< 0.01 for irradiated 0% FLC vs. irradiated 10% and 20% FLC.

Additionally, lipid peroxidation indicated by MDA levels in the BAL fluid were also significantly (*p*<0.01) depressed with the FLC diet (Figure 6B). Specifically, while radiation induced a robust 5-fold increase over non-irradiated mice on the control diet (*p*<0.05), levels remained low (comparable to non-irradiated levels) in BAL fluid from mice fed FLC diets.

### Dietary FLC mitigated lung inflammation induced by a single fraction of thoracic radiation

Radiation pneumonopathy is in part defined as an increase in inflammatory cells within the lungs. An early influx of cells wreaks havoc in the parenchyma and contributes to late collagen deposition and fibrosis. To test if dietary FLC is as effective a mitigator of radiation induced lung injury as whole grain FS, shown in our previous studies [13,21,22], we measured total WBC and neutrophils (PMN) cells/ml of bronchoalveolar lavage fluid (BAL) in irradiated mice fed the test diets given at defined time points post-XRT. BAL white blood cells per ml/ BAL fluid obtained from non-irradiated mice fed 0% FLC, 10% FLC, and 20% FLC totaled approximately 50,000 cells. In contrast, irradiated mice fed control 0% FLC diet had 125,000 cells/ml BALF. Cell numbers were significantly reduced (*p*<0.01) in irradiated mice fed 10% FLC diets 24 hours and 48 hours post-XRT exposure (Figure 7A) compared to irradiated mice fed control (0% FLC) diet. Notably, mice fed 10% and 20% FLC diets 48 hours post-XRT displayed significantly (*p*< 0.05) decreased inflammation after irradiation with reduced PMN cells/ml BALF compared to their irradiated counterparts fed 0% FLC diet (Figure 7B). Importantly, irradiated mice fed 10% and 20% FLC 24 and 48 hours post-XRT showed a significantly lower (*p*<0.05) influx of inflammatory cells/ml BAL fluid compared to irradiated control mice fed 0% FLC sacrificed at 16 weeks, reinforcing the concept that early intervention with a radiation mitigating agent is preferable in order to yield the greatest long-term benefits.

**Figure 7:** **Evaluation of lung inflammation in mice at 16 weeks post-XRT.** Mice were pre-fed 0% FLC for 72 hours prior to single fraction thoracic X-ray radiation therapy (13.5 Gy). Following XRT exposure, mouse cohorts (n=15) were fed 10% FLC or 20% FLC diets initiated 24, 48, or 72 hours post-XRT. Control-fed mouse cohorts remained on 0% FLC diet throughout the course of the study. Mice were sacrificed at 16 weeks post-XRT and bronchoalveolar lavage (BAL) fluid was collected. **Panel A**: Total WBC counts in BAL fluid. Data is represented as mean ± SEM. *p≤ 0.01 for irradiated 0% FLC vs. Irradiated 10% FLC. **Panel B**: Total PMN cells in bronchoalveolar lavage (BAL). Data is represented as mean ± SEM. *p< 0.05 for irradiated 0% FLC vs. irradiated 10% and 20% FLC (+48 hours).

### Dietary FLC protected against fibrosis after a single fraction of thoracic radiation

Semi-quantitative analyses using an established scale of fibrosis/inflammation as previously described in Lee, et al. 2009 [21] on Trichrome-stained sections was performed to assess the extent of radiation fibrosis within murine lung tissue. Representative samples of lungs from mice fed test diets are shown in (Figure 8) where Trichrome staining revealed higher collagen deposition in irradiated murine lungs on 0% FLC diet (Panels A-C) as compared to 10% (Panels D-F) and 20% FLC diets (Panels G-I). This was supported by decreased alveolar congestion and edema.

**Figure 8:** **Histological evaluation of lung fibrosis at 16 weeks post -XRT.** Mice on control diet (0% FLC) were exposed to a single fraction thoracic X-ray radiation therapy (13.5 Gy). Following XRT exposure, mouse cohorts (n=15) were switched to 10% FLC or 20% FLC diets that were initiated 24, 48, or 72 hours post radiation exposure while control-fed mouse cohorts remained on 0% FLC diet throughout the course of the study. Lungs were harvested at 16 weeks post-XRT and processed for Trichrome staining to evaluate collagen deposition and fibrosis. Representative lung sections stained with Trichrome are shown on **Panels A-C**: representing 0% FLC, **Panels D-F**: representing 10% FLC and **Panels G-I**: representing 20% FLC. (Magnification 400X).

Results of histopathological staining for collagen were reinforced via quantification of the hydroxyproline content in the lungs. Baseline levels of hydroxyproline under all dietary conditions without irradiation are shown in Figure 9A (hatched bars). Significant production of lung hydroxyproline was induced in irradiated mice fed control 0% FLC diet (Figure 9A, hatched). Levels increased from baseline 89.32±6.05 μg per lung to 149.24±6.03 μg per lung respectively in mice fed 0% FLC. Lung tissue of irradiated mice fed 10% FLC 24 hours post-XRT displayed significantly (*p≤*0.001) decreased hydroxyproline content compared to control diet, with 110.67±5.79 μg/lung. Significant reductions (*p≤*0.01) of hydroxyproline content with feeding 20% FLC at 48 and 72 hours post-XRT compared to control-fed mice was also noted. Lastly, significant reduction (*p*<0.05) in hydroxyproline content was also seen with 20% FLC at 24 hours post-XRT compared to control.

**Figure 9:** **Determination of fibrotic changes in murine lungs at 16 weeks post-XRT.** Mice were pre-fed 0% FLC for 72 hours prior to single fraction thoracic X-ray radiation therapy (13.5 Gy). Following XRT exposure, mouse cohorts (n=15) were fed 10% FLC or 20% FLC diets initiated 24, 48, or 72 hours post-XRT. Control-fed mouse cohorts remained on 0% FLC diet throughout the course of the study. Lungs were harvested at 16 weeks post-XRT. **Panel A**: Evaluation of hydroxyproline content in lungs. Data is represented as mean ± SEM. *p< 0.05 for irradiated 0% FLC vs. irradiated 10% FLC and 20% FLC, #*p*≤ 0.01 for irradiated 0% FLC vs. irradiated 20% FLC (+48 and +72 hours), $*p*≤ 0.001 for irradiated 0% FLC vs. irradiated 10% FLC (+24 hours). **Panel B**: Fibrotic Index (range=0-4) scoring. Data is represented as mean ± SEM. *p< 0.05 for irradiated 0% FLC vs. 10% FLC (+48 hours).

Along with hydroxyproline analysis, histopathological scoring (Fibrotic Index Score Figure 9B) performed by a lung pathologist (CCS) blinded to the study design, demonstrated that feeding 10% FLC 48 hours post-XRT led to significantly decreased (p<0.05) extent of pulmonary fibrosis after a single fraction of 13.5 Gy thoracic radiation. Overall, providing FLC post-XRT showed dose response and time response curves. Although not statistically significant at all points, Figure 9B shows that the highest dose of FLC at the earliest time point after irradiation displayed the lowest fibrotic index score.

### Flaxseed Lignan Component Modifies the Expression of Regulatory Cytokines

Cytokine and chemokine levels in BAL fluid post-irradiation signify activation of inflammatory pathways that are involved in the pathogenesis of radiation-induced lung injury. We anticipated that the lignan component in flaxseed would mitigate activation of the inflammatory pathway. As seen in Table 1, 13.5 Gy thoracic radiation significantly (*p*<0.01) increased key cytokine levels in BAL fluid when compared to non-irradiated controls. This increase in the concentration of certain cytokines, such as FGF-basic, IL-12, and VEGF, was significantly (*p*<0.05) mitigated by FLC, irrespective of when the diet was initiated. Overall cytokine and chemokine levels were reduced or even undetectable in the BAL fluid of irradiated mice fed FLC as compared to control counterparts.

**Table 1:** BAL fluid cytokine levels in mice 16 weeks post-XRT

	**Cytokine values (pg/ml) (mean ± SEM)**						
	**FGF-basic**	**IL-5**	**IL-6**	**IL-12 (p40/p70)**	**KC**	**MCP-1**	**VEGF**
***No XRT (13.5 Gy)***							
0% FLC	ND^1^	4.6 ± 0.6	3.7 ± 0.2	3.2 ± 1.2	ND^1^	3.3 ± 0.9	10.9 ± 1.5
10 % FLC	ND^1^	2.3 ± 0.6^a^	2.6 ± 0.8	0.2 ± 0.1	ND^1^	3.9 ± 1.0	8.5 ± 1.8
20% FLC	ND^1^	2.1 ± 0.3^a^	2.4 ± 0.6^a^	ND^1^	ND^1^	2.7 ± 0.8	5.7 ± 0.5^a^
***XRT (+24 Hours)***							
0% FLC + 13.5 Gy	52.5 ± 5.5^b^	15.3 ± 5.3	129.0 ± 86.6	114.5 ± 24.5^b^	261.8 ± 52.6	77.9 ± 39.7	47.2 ± 5.0^b^
10% FLC + 13.5 Gy	55.3 ± 5.4	5.2 ± 0.9	ND^1^	73.4 ± 25.9	18.1 ± 4.4	27.2 ± 0.7	52.1 ± 9.3
20% FLC + 13.5 Gy	36.0 ± 6.4	10.7 ± 4.5	49.1 ± 22.3	91.1 ± 21.4	ND^1^	29.1 ± 0.9	38.4 ± 3.3
***XRT (+48 Hours)***							
0% FLC + 13.5 Gy	52.5 ± 5.5	15.3 ± 5.3	129.0 ± 86.6	114.5 ± 24.5	261.8 ± 52.6	77.9 ± 39.7	47.2 ± 5.0
10% FLC + 13.5 Gy	61.7 ± 4.8	2.1 ± 0.3^c^	38.4 ± 12.8	6.7 ± 2.3^c^	ND^1^	26.8 ± 1.5	7.2 ± 3.0^b^
20% FLC + 13.5 Gy	37.5 ± 8.6	7.3 ± 3.6	132.3 ± 75.0	83.7 ± 34.6	ND^1^	28.2 ± 1.7	39.7 ± 11.8
***XRT (+72 Hours)***							
0% FLC + 13.5 Gy	52.5 ± 5.5	15.3 ± 5.3	129.0 ± 86.6	114.5 ± 24.5	261.8 ± 52.6	77.9 ± 39.7	47.2 ± 5.0
10% FLC + 13.5 Gy	35.6 ± 11.2	13.7 ± 7.6	369.7 ± 241.7	88.1 ± 32.5	425.7 ± 141.9	82.5 ± 49.9	33.0 ± 10.5
20% FLC + 13.5 Gy	34.8 ± 8.8	2.3 ± 0.8^c^	ND^1^	22.7 ± 11.8^c^	ND^1^	23.1 ± 0.7	30.2 ± 9.5

^1^ND = Not Detectable in Assay.

a = *p*≤0.05 for non-irradiated 0% FLC vs. non-irradiated 10% FLC and 20% FLC.

b = *p*<0.01 for non-irradiated 0% FLC vs. irradiated 0% FLC.

c = *p*<0.05 for irradiated 0% FLC vs. irradiated 10% FLC and 20% FLC.

Mice were pre-fed 0% FLC for 72 hours prior to single fraction thoracic X-ray radiation therapy (13.5 Gy). Following XRT exposure, mouse cohorts (n=15) were fed 10% FLC or 20% FLC diets initiated 24, 48, or 72 hours post-XRT. Control-fed mouse cohorts remained on 0% FLC diet throughout the course of the study. Mice were sacrificed at 16 weeks post-XRT and bronchoalveolar lavage (BAL) fluid was collected. BAL cytokine analysis was performed and data is represented as mean ± SEM. a= *p*≤0.05 for non-irradiated 0% FLC vs. non-irradiated 10% FLC and 20% FLC, b= *p*<0.01 for non-irradiated 0% FLC vs. irradiated 0% FLC, and c= *p*<0.05 for irradiated 0% FLC vs. irradiated 10% FLC and 20% FLC.

Positivity for TGF- beta1 in lung tissues at 16 weeks post radiation exposure was assessed using immunohistochemistry (Figure 10A) followed by image analysis to quantify the extent of positivity (Figure 10B). Staining of lung sections for a representative mouse cohort (diet added 24 hours post XRT) revealed a robust 2.5-fold increase in staining intensity for TGF-beta1 in irradiated lungs fed control diets as compared to non-irradiated controls. Importantly, TGF- beta1 positivity in lungs from irradiated mice fed FLC diets remained at baseline levels (*p*<0.03) (Figures 10B).

**Figure 10:** **Immunohistochemical detection and quantification of TGF-beta1 in lung at 16 weeks post –XRT.** Mice on control diet (0% FLC) were exposed to a single fraction thoracic X-ray radiation therapy (13.5 Gy). Following XRT exposure, mice were switched to 10% FLC or 20% FLC diets that were initiated 24 hours post radiation exposure while control-fed mouse cohorts remained on 0% FLC diet throughout the course of the study. Lungs were harvested at 16 weeks post-XRT, paraffin embedded and immunostained for TGF beta1; brown staining (**Panel A**). Representative lung sections are shown In **Panels a-b:** representing 0% FLC, **Panels c-d:** representing 10% FLC and **Panels e-f**: representing 20% FLC. Sections were counterstained with methyl green. (Magnification 400X). Quantification of TGF-beta1 positivity (**Panel B**) was made using the Aperio image analysis system. #p<0.03 as compared to irradiated 0% FLC.

## Discussion

We have shown here for the first time that the lignan component of flaxseed, enriched in the lignan SDG, administered within just 24–72 hours post-thoracic radiation enhanced survival and mitigated the chronic lung injury induced by XRT. We determined that FLC-supplemented diet mitigated the deleterious effects of XRT by: 1) improving blood oxygenation levels, 2) decreasing lung injury by lowering BAL protein levels, 3) reducing pulmonary fibrosis by decreasing collagen content and TGF-beta1 levels of lung tissues, 4) reducing lung inflammation by decreasing WBC influx into the airways and most importantly, 5) reducing oxidative tissue damage as shown by decreased protein nitration in lung tissue and lipid peroxidation in BAL fluid 6) improving overall animal survival.

Radiation-induced injury to adjacent normal tissue is a notable sequelae of ionizing radiation exposure [7]. Our results indicated that XRT-induced lung inflammation and impaired blood oxygenation (decreased SaO2) were improved with 10 and 20% FLC diet when initiated after XRT. Vujaskovic and coworkers [7,34] have shown that severe hypoxia develops months post an initial radiation exposure of lung tissues. Such hypoxia resulted from the development of a cascade of events leading to lung injury. Improved blood oxygenation of all FLC-fed mouse groups may lead to decreased levels of tissue hypoxia and may therefore explain the mitigation of adverse radiation effects even when diets are initiated post challenge. Decrease of radiation-induced lung inflammation by a mitigator was first shown by our group in whole grain FS [22]. This is the first report that FLC mitigated pulmonary inflammation when given hours post initial XRT challenge.

A major feature of radiation pneumonitis is a considerable increase in alveolar protein accumulation, an indicator of increased vascular permeability and direct lung injury [35]. Radiation damages resident lung cells that subsequently release inflammatory cytokines and chemokines that recruit inflammatory cells to that area of injury while priming the immune system in a cyclic-feedback loop [36]. BAL protein levels are a direct and reliable measure of lung injury, translating into actual tissue damage while lung inflammatory cell markers (although useful) serve as a surrogate measure of inflammation and not injury directly [34]. Our results show significant mitigation of lung injury in all the experimental FLC diet fed groups, regardless of the timing of diet initiation. This may be attributed to decreased inflammatory cell influx and membrane oxidation in FLC-supplemented mice. In addition, we noted decreased oxidative tissue damage in FLC-fed mice, as evidenced by the tissue levels of nitrotyrosine and MDA levels in the BAL fluid. Antioxidant agents capable of decreasing nitrotyrosine have also been shown by others to be protective in radiation lung damage [37]. We first reported [22] that whole grain FS was able to mitigate physiological lung injury from radiation *in vivo*. We now are the first, to our knowledge, to report that FLC demonstrates similar *in vivo* beneficial properties as the whole grain, strongly suggesting that FLC contains the key bioactive radiation mitigator found in FS.

Radiation pneumonitis chronically evolves into fibrotic changes within lung tissues as a late phase of the radiation exposure response mechanism [38]. We have shown that whole grain FS was protective against experimental radiation fibrosis [21] and as a mitigator of late radiation induced lung changes after one dose of thoracic XRT [22]. Our current study showed for the first time that via FLC, fibrotic processes associated with high TGF-beta1 levels in lung tissues can be blunted even when the protective agent is given post-radiation damage, i.e., as a radiation mitigator. Notable benefits including quantitative and qualitative physiologic and histopathologic endpoints from the therapeutic use of FLC diet when initiated at 24, 48, 72 hours posts XRT demonstrate that FLC is a highly bioactive radiation mitigator. However, FLC-mediated decline in both lung hydroxyproline levels and fibrotic index were more prominent when diet was started preventively, i.e., 3 weeks prior to XRT. This suggests that further development or modification of the bioactive component(s) of FLC has the potential to further improve the properties of this novel dietary radiation mitigator.

Regulatory cytokines and chemokines play a significant role in the inflammatory response implicated in radiation induced lung injury. The detection of pro-inflammatory cytokines, such as IL-6 and IL-12, in the BAL of irradiated mice at 4 months post-XRT signifies a chronic and sustained inflammatory state that occurs post-irradiation. This heightened level of inflammation may play a significant role in the development of pulmonary fibrosis. We have previously reported that whole grain flaxseed when given as radiation mitigator reduces the concentration of pro-inflammatory cytokines present in BAL fluid [22]. Based on our current findings, this reduction in BAL cytokine levels may be conferred by the lignan component in whole grain flaxseed.

Lung lavage has been advocated as a possible countermeasure to remove radionuclides inhaled after detonation of an RDD [39,40]. However, this seems impractical since multiple lavages may be required for efficient removal of radionuclide burden using an invasive procedure with inherent risks and a requirement of anesthesia. Alternatively, a plethora of synthetic and natural compounds are being evaluated with the intent of mitigating radiation damage [19]. Agents are being developed that target inflammatory cell recruitment, free radical production, cell death, cytokine and growth factor expression, and other cell functions [5,10,41]. While Amifostine is the only FDA approved cytoprotective radiation mitigator its use has been associated with significant systemic toxicity [19]. Furthermore, many of the compounds that had offered cellular radioprotection *in vitro* have not demonstrated pre-clinical *in vivo* efficacy, as summarized in a recent review by Williams et.al. [10]. Despite much progress, the search for an effective and safe radiation mitigator with clinical usefulness has yet to be identified.

An ideal radiation mitigator should be safe, effective, have an easy route of administration and a long shelf-life. The bioactive flaxseed lignan complex (FLC) enriched in the phenolic secoisolariciresinol diglucoside (SDG) has become a topic of study because of its anti-inflammatory, antioxidant and anti-fibrotic attributes most notably in models of thoracic radiation induced acute and chronic lung injury [20]. Importantly, prolonged FLC administration in our animal models has not led to any significant toxicity. This is a critically important feature, since administering a radiation mitigator that possessed even mild toxicity in healthy individuals to a large population following radiation exposure could lead to severe toxicity in individuals with additional medical co-morbidities. Furthermore, FLC has a long, stable shelf life and is easy to administer orally at an affordable price. We therefore posit that FLC may be an effective, safe and cost-effective mitigator of radiation damage.

It is evident from our results that FLC diet given within 24–72 hours after thoracic radiation exposure has benefits in terms of morbidity and mortality. Improvement of survival using antioxidants such as N-acetyl-Cysteine (NAC) or mitochondrial-targeted small molecule radiation damage mitigators have been shown in mouse models of abdominal irradiation [42] or total body irradiation [43] respectively. To our knowledge our study is the first to report that FLC served this same purpose improving survival of animals in an experimental model of thoracic radiation damage without any significant side effects or difficulties in oral administration, often associated with NAC given the unpleasant smell of its oral formulation.

In summary, we have evaluated a non-toxic, widely available dietary phenolic compound that yielded late protective benefits after lung exposure to radiation. We have studied the beneficial properties of whole grain FS in the past. Here for the first time we demonstrated that FLC surpassed whole grain FS in its antioxidant, anti-inflammatory and anti-fibrotic mitigation properties when administered after thoracic XRT. FLC altered immediate XRT-induced markers of lung damage, creating a radioprotective milieu post-XRT, and provided high levels of circulating antioxidants from the continued metabolism of its bioactive lignans. Our long-term goal is to provide that long awaited, safe to consume, easy to administer, inexpensive compound for large populations in either the post-therapeutic radiation scenario or post-radiologic terrorism (dirty-bomb) event. That compound is the flaxseed lignan complex.

## Conclusion

There is an unmet need to identify a radiation-mitigating agent that is effective in blunting adverse radiation effects to the lung, while being at the same time inexpensive, non-toxic, and easy-to-deliver to the wider population that may include people with diverse underlying medical conditions. Our findings that the lignan component in flaxseed is a potent mitigator of radiation induced lung injury in a preclinical model of radiation pneumonopathy signifies the potential for the use of FLC in clinical settings. In the past, we have shown that whole grain flaxseed, when given at various time points post-XRT, was able to blunt the negative effects to the lung of acute radiation exposure. Early intervention with the lignan component of flaxseed proves to be equipotent in mitigating radiation-induced lung injury by decreasing inflammation, cytokine release, TGF-beta1 tissue levels, oxidative tissue damage and subsequent collagen deposition post-XRT, while improving important parameters such as oxygenation and overall survival that are implicated in improved clinical outcomes.

## Abbreviations

BALF: Bronchoalveolar lavage fluid; ED: enterolactone; EL: enterodiol; FI: Fibrotic Index; FS: Flaxseed; FLC: Flaxseed Lignan Complex; H&E: Hematoxylin and eosin; IR: Irradiation; MDA: Malondialdehyde; PMN: Polymorphonuclear leukocyte; ROS: Reactive oxygen species; SARRP: Small animal radiation research platform; SDG: Secoisolariciresinol diglucoside; SEM: Standard error means; WBC: White blood cells; XRT: X-ray Treatment.

## Competing interests

The authors declare that they have no competing interests.

## Authors’ contributions

MCS: Designed the study and individual experiments, analyzed data, wrote the manuscript and supervised project and lab personnel; JBT: Analyzed data, assisted in writing of the manuscript, and performed final editing; ST: Assisted with animal experiments and manuscript preparation; SH: performed all the irradiation procedures; RP: Performed animal experiments, biochemical assays and conducted data analysis; FD: Assisted with pulse oximetry; EA: Conducted animal experiments and tissue analyses; CCS: Performed pathology assessment of histological specimens; KAC: Provided consultation on data analysis; TB and SGC assisted with the TGF- beta evaluation in tissues. All authors read and approved the final manuscript.

## Pre-publication history

The pre-publication history for this paper can be accessed here:

http://www.biomedcentral.com/1471-2407/13/179/prepub
